This article has been retracted.

# Design of Optimal Scheduling Model for Emergency Medical Supplies by Blockchain Technology

**DOI:** 10.1155/2022/4608761

**Published:** 2022-02-18

**Authors:** Yan Zhao

**Affiliations:** College of Management, China University of Mining and Technology, Xuzhou, Jiangsu, China

## Abstract

The study aims to explore the scheduling plan for the emergency of blockchain technology in the medical industry. Network security architecture for medical supplies management based on the Hyperledger Fabric optimized consensus mechanism is established by studying the characteristics of blockchain technology and its data structure composition. The supply chain model for medical device scheduling based on intelligent contracts is selected for the particularity of the nature and shape of medical devices in medical supplies. Ant colony algorithm is used to solve it. Case analysis and verification results show that the improved Hyperledger Fabric consensus mechanism has better security performance. Under the condition of 10,000 transactions, the probability of an attacker with the optimized consensus mechanism successfully controlling the transaction is only 7.2%. The optimized solution is about 50% higher than the original solution in terms of transaction processing speed. Over 1000 transactions, the transaction latency optimization rate is more than doubled. The total order completion time of the medical device scheduling model adopted by the intelligent contract is 26.3% higher than the historical service time of 19 days. The performance of the medical emergency material scheduling program that is added to the supply chain technology is better.

## 1. Introduction

The handling of medical emergencies is related to everyone's life and health. For example, the rapid coronavirus disease 2019 (COVID-19) outbreak in the past two years has spread to the world [1]. The efficiency and accuracy of medical supplies dispatching in such incidents require close collaboration and cooperation between the medical staff of various medical institutions and personnel of multiple institutions, such as logistics systems in order to minimize the risk of human life safety [2]. The characteristics of decentralization, transparency, autonomy, and nontameability of blockchain technology can keep the quantity, location, and delivery status of medical supplies under real-time control during the medical supplies dispatching process. It can provide timely adjustment plans according to the development status of medical emergencies [3–5]. Therefore, the establishment of such a log scheduling system with the blockchain as the global control gives the platform the ability to trace any form of data modification, which can ensure that any data modification operation is transparent to all personnel of the medical institution participating in the collaboration. It can ensure the integrity of data during the transportation of medical supplies, thereby establishing a trust relationship between multiple agencies involved in the prevention and control of public emergencies. Meanwhile, it can also greatly reduce the communication costs and conflicts caused by mutual distrust and improve the efficiency of material scheduling [6].

Regarding the application of blockchain technology in the scheduling of medical supplies, scholars have also achieved a lot of research results. The huge amount of data in the healthcare system makes it difficult to ensure safety and diagnostic procedures. In order to solve these problems, Sammeta and Parthiban [7] developed a new ultrazipper blockchain to support safe medical data management using deep learning diagnostic models. The presented model involves different stages of operation, such as encryption, optimal key generation, blockchain-based super-blockchain security data management, and diagnosis. The integration of the Internet of Things (IoT) in the medical system can support medical events, such as real-time diagnosis, remote patient monitoring, and real-time drug prescriptions. However, the integrity and confidentiality of medical information on the Internet of Medical Things (IoMT) platform is still one of the controversies leading to medical service issues. Ogundokun et al. [8] proposed an Encryption-Stegno model to ensure medical information about the IoMT environment. In response to the Acquired Immune Deficiency Syndrome (AIDS) epidemic, stakeholders such as clinicians, community advocates, and researchers have used various forms of technology to alleviate the crisis. Garett and Young [9] pointed out that blockchain was an emerging technology that originated from cryptocurrency. The function of the blockchain is very suitable for working in HIV. Its ability to safely transmit information and interact makes it a potentially useful tool. It can incorporate research and practice related to stigmatized diseases such as HIV, which require methods to maintain a high degree of security and confidentiality. There are many researches on the application of blockchain technology in the medical industry, but there are few studies in the field of medical material dispatching. The research on the dispatch of emergency supplies for medical emergencies can fill this research gap.

Using the methods of literature research and model verification, the study discusses the application of blockchain technology in medical material distribution. The innovation is that the optimized Hyperledger Fabric mechanism is adopted. The security, running speed, and transaction delay of the medical material dispatching network platform are improved. Ant colony algorithm is used to optimize the supply chain model for medical device scheduling logistics. Compared with similar studies in other related fields, this model can obtain shorter order completion time, and the transaction processing speed and transaction optimization rate have been greatly improved. The study is structured as follows.  Section 1 describes the application background and current research status of blockchain technology in medical emergencies.  Section 2 introduces the security analysis of medical material management based on the Hyperledger Fabric consensus mechanism.  Section 3 compares and analyzes the corresponding research results given by the research method in Section 2, and Section 4 is the research conclusion.

## 2. Materials and Methods

### 2.1. Blockchain Technology and Its Data Structure

Blockchain technology is a decentralized distributed database integrated by multiple technologies. It uses Distributed Ledger Technology (DLT), which is a decentralized recording method [10]. There is no need to establish a trust relationship between each node of the blockchain. All node members in the blockchain can participate in data maintenance. Every node participating in the maintenance can obtain a complete copy of the blockchain data. Therefore, the blockchain is often described as a distributed ledger in which all nodes participate in the accounting records [11]. Each participant has their own complete copy of the ledger. Compared with traditional databases that emphasize centralization, blockchain technology maintains the characteristics of decentralization, transparency, autonomy, and immutability [12].

The characteristic of decentralization means that all nodes in the blockchain have an equal relationship, and there is no trust center node. All nodes jointly maintain the data on the blockchain, which is the most fundamental feature of blockchain technology. Transparency is the basis for ensuring mutual trust among system nodes [13]. All update operations of nodes in the entire network are open and transparent to other nodes. All nodes can obtain any data and update records at any location in the blockchain at any time when needed [14]. No human intervention is required. All of its behaviors are autonomous, and only a predetermined algorithm determines how to operate. The cryptography technology in the blockchain can ensure that all data on the blockchain cannot be modified but can only be added. Because the cost of modifying the data on the blockchain is very high, this ensures that the blockchain data cannot be tampered with [15]. Blockchain architecture usually consists of a data layer, network layer, public awareness layer, incentive layer, contract layer, and application layer [16]. The data structure of the Bitcoin block is shown in Figure 1:

### 2.2. Recent Research Work on Blockchain Technology

In recent years, blockchain-based decentralized cryptocurrencies have attracted a lot of attention. Bitcoin is the first blockchain application, which has achieved great success and promoted more development in this field. However, the development of Bitcoin has encountered performance problems of low throughput and high transaction latency. Other cryptocurrencies based on proof-of-work also have these shortcomings, leading to more concerns about the scalability of the blockchain. Zhou et al. [17] tried to cover the existing extended blockchain solutions and classify them by level. In addition, they compared different methods and listed some potential directions for solving blockchain scalability issues. Various innovative applications are growing exponentially, such as smart agriculture, innovative healthcare, supply chain, logistics, commerce, tourism and hotels, energy management, etc. However, open channels for all applications, security, and privacy are the main issues. However, many security solutions and standards have been proposed to enhance the security level of intelligent applications. The existing solutions are either based on a centralized architecture or have high computing and communication costs. In addition, most existing security solutions only focus on a few aspects and fail to address the issues of scalability, robustness, data storage, network latency, immutability, and traceability. Blockchain technology has become one of the solutions to these problems. Based on these facts, Bodkhe et al. [18] conducted a systematic analysis of various blockchain-based solutions and their applicability in diverse industry 4.0-based applications. Many experts analyzed the potential applications of blockchain technology in different aspects of markets, institutions, or government organizations. In the brief history of blockchain, the use of blockchain has made incredible achievements. These aspects' sheer number and complexity may make it difficult to solve the blockchain problem. Nanayakkara et al. [19] found that the structure of blockchain and modern cloud edge computing are essential for new participants to realize the widespread adaptation and development of blockchain technology. The use of public and open-source codebases and tools will help ensure that the full potential is acknowledged of the blockchain.

### 2.3. Security Analysis of Medical Supplies Management Using Hyperledger Fabric Consensus Mechanism

Hyperledger Fabric network platform, as a kind of blockchain consensus mechanism, is an open and open-source project. Although the Hyperledger Fabric network platform is also decentralized like blockchain technology, the status of nodes in its network is different. Ordinary nodes must be authorized and authenticated by special nodes in the network before they can be added, which can reduce resource consumption while increasing transaction processing speed [20–22]. Applying it to the management part of material scheduling for medical emergencies can ensure data security and transmission speed in the material scheduling process. The original consensus mechanism of Hyperledger Fabric is shown in Figure 2:

First, the client will generate a proposal. Then, the proposal is sent to the endorsing node. The proposal has the on-chain code that needs to be executed, that is, the smart contract and some other information that contains the signature carried by the client and the time stamp of the proposal generation. The endorsement node verifies whether the proposal is sent by the authenticated client by sending the signature in the proposal from the client. If not, the endorsing node will terminate the transaction. The result of the execution generates a set of read and write sets using the current ledger status. When there are multiple sorting nodes in all ledgers, the system will automatically call the Kafka cluster to sort transactions according to certain rules. There are some problems with this mechanism: after the transaction speed is increased, the existence of some key nodes will cause a certain “centralization” problem in the entire system due to the unequal relationship between nodes. In order to improve the security and performance of the Hyperledger Fabric consensus mechanism, a dynamic random method is used to determine the identity of the endorsing node. The optimized Hyperledger Fabric consensus mechanism is shown in Figure 3:

Since the endorsement node of the optimized scheme is randomly selected by using a verifiable random function, this virtually strengthens the security and privacy of the node and reduces the possibility of the node being attacked. The use of a verifiable random function can reduce the possibility of a fixed number of nodes always serving as endorsing nodes, which reduces the degree of centralization of endorsing nodes. Since the optimized node is no longer fixed because of the endorsement node, the probability of being attacked successfully will be reduced, which can improve the security of the system. Attacking hackers want to successfully attack and control a candidate endorsing node. Trying to use this as an opportunity to destroy the entire transaction is almost impossible. Because the system needs to select only one node during the attack, and this node happens to be controlled by the adversary. The probability of occurrence of this situation is shown in the following:

(1) $$\begin{array}{c} \text{pr}=\frac{1}{n}\overset{1}{\underset{n}{c}}{\left(1-\lambda \right)}^{n-1}={\left(1-\lambda \right)\lambda }^{n-1}. \end{array}$$

*λ* represents the present threshold for selecting endorsement nodes, and *n* represents the number of peer nodes included in the candidate endorsement node set. Assuming that the number of candidate endorsement nodes is 10, the threshold is 0.4. Then control an endorsement node, and the probability that the attacker can interfere with the transaction is as follows:

(2) $$\begin{array}{c} {\text{pr}}_{i}=\left\{\begin{array}{c} \overset{i}{\underset{k}{c}}{\left(1-\lambda \right)}^{i}{\left(\lambda \right)}^{n-i},\;0<i\leq k,\\ \overset{i-k}{\underset{n-k}{c}}{\left(1-\lambda \right)}^{i}{\left(\lambda \right)}^{n-i},\;k<i<2k. \end{array}\right) \end{array}$$

*pr*_*i*_ represents the probability that the adversary can interfere with the transaction. *k* represents the number of endorsement nodes. *λ* represents the required threshold for selecting endorsement nodes set in advance. *n* represents the number of peer nodes contained in the candidate endorsement node set. The probability of an attacker who successfully interferes with the transaction by controlling *k* endorsing nodes is shown in the following:

(3) $$\begin{array}{c} \text{pr}=\sum_{i=1}^{n}{pr}_{i}. \end{array}$$

When facing the same transaction, many clients have different random numbers, and their endorsement nodes are also different. Endorsement nodes that are not selected can simultaneously endorse other clients. This parallel processing mode can speed up transaction processing. In addition, from the moment a client initiates a transaction until the transaction is recognized by the entire network, the process of endorsing the transaction by the candidate endorsing node may increase the transaction process time and cause transaction delay. There are usually some problems in applying this improved scheme to the existing medical material dispatching platform. The network deployment topology is shown in Figure 4. The disadvantages of centralized data storage are obvious. All electronic data are stored in a centralized central server. Once this server is attacked by hackers, it will face data leakage and malicious tampering of data. This will cause devastating consequences and immeasurable economic losses to all medical material platforms. If affected by natural disasters, the entire system will face collapse and system security will be low. As enterprise business expands and the number of orders increases, platform data will show explosive growth. This requires the establishment of a central server with stronger processing capabilities, and the centralized storage requires a huge amount of funds to be used for third-party centralized organizations to ensure the smooth operation of the system, and the cost is high. In addition, traditional electronic documents will go back and forth along the entire supply chain with the materials, requiring a lot of complicated operations. In order to ensure the safe operation of the system, a centralized third-party organization is often required to assist in the certification, which invisibly leads to relatively low efficiency of all processes. Applying the above-mentioned improvement scheme to this kind of medical material dispatching system can improve these problems to a great extent.

The application of blockchain technology in the material scheduling platform, and the private chain operation in the early stage, can not only ensure the security and authenticity of data but also improve the efficient collaboration of various units within the enterprise in the material fulfillment process. Suppliers and other external units use the “real-name identity authentication + service agreement” method to achieve business linkage through application identity access management and quick access to the platform. The core database is placed in the company's information and communication computer room, and the database is used to store core business data.

In the mid-term, the system will build a larger range of alliance chains in conjunction with other organizations or authorities on the basis of the existing private chain. Meanwhile, the consortium chain can set an admission mechanism for the joining nodes, and the nodes can perform limited queries through the Application Programming Interface (API) [23] opened by the blockchain. The expanded network topology is shown in Figure 5:

In the later period, the robustness and stability of the entire platform is considered. If conditions permit, the platform will eventually adopt the Kafka cluster deployment mode. Among them, the order node will also be deployed in a cluster. In order to further ensure the immutability and authority of the consortium chain, by gradually increasing the members of the consortium chain, if conditions permit, at least one public trust institution shall be introduced as a consortium member to ensure the credibility of the consortium chain. Therefore, the final network topology is shown in Figure 6:

According to the final network structure, the minimum server configuration requirements are: a server with expansion requirements. It requires a 4-core Central Processing Unit (CPU), a memory of 4G, a hard disk capacity of 500G, and an operating system of Centos7.4. There are three servers each, ZooKeeper, Kafka, and Order in this configuration. To ensure consistent blockchain technology, superior stability and performance, the minimum hardware configuration requirements for the added node are: 1 server, Centos7.4 operating system, 4-core CPU, memory at least 4G, and hard disk capacity above 1T.

System performance is tested and safety is tested. Ten candidate endorsement nodes are selected, and 5 endorsement nodes successfully attacked by the adversary. Golang1.9 is used by the platform, and the crypto package in Golang is used to verify random functions. The curve-p256 elliptic curve is adopted. The hash function is sha-256, which can better show the advantages of the optimization scheme. The transaction speed is tested: the present number of candidate endorsement nodes is 10, and the threshold is 0.4. When 1, 10, 100, and 1000 transactions are initiated, the original plan and the optimized plan are compared with the average time it takes to successfully process each transaction in the medical material platform.

### 2.4. Construction of Smart Contract Model of Medical Device Dispatching Supply Chain

Medical emergencies often carry great safety risks. Therefore, timely measures such as emergency preparations, monitoring, prediction, early warning, reserve, and on-site disposal shall be taken to prevent possible factors that may cause public health emergencies, and to prevent the emergence of public health emergencies. The control of public health emergencies requires a certain degree of timeliness. As a kind of medical supplies, medical equipment has many problems in the dispatching process. Smart contracts are codes that are stored, verified, and executed on the blockchain and are a way of spreading through information channels. It completes the business logic assigned by the user according to the preset instructions to verify and execute the computer protocol of the task.

Because of the different types of medical devices and different models and sizes, biological and chemical reactions may occur between each other during the scheduling process. Therefore, there are higher requirements for storage and transportation conditions, logistics environment and timeliness, tracking and monitoring of the entire logistics, and management capabilities of logistics service providers. In addition, the lack of close cooperation among enterprises in the medical device logistics service supply chain, the lack of large-scale medical device logistics service integrators, and the lack of unified data management norms and standards for data collection among logistics enterprises have led to some links in the logistics service supply chain. “Information distortion,” resulting in poor timeliness of product traceability. Smart contracts can provide smart carriers for all kinds of information such as accounting, transactions, assets, funds, etc. Using the form of blockchain data code to spread across the network, after the security key and the auxiliary confirmation of the front and rear blocks, each node is stored in a time series information. This technology can improve information fraud, tampering, and even deletion. It has the advantages of efficient real-time update, accurate execution, reduced human influence, decentralization, and lower operating costs.

The smart contract technology is used in the supply chain of medical equipment logistics scheduling, and the process design of the smart contract model is shown in Figure 7. Many logistics service providers can perform operational services in the supply chain, and these operational services are arranged in order as a service process. In the design of smart contracts, the state change mechanism is one of the core mechanisms of logistics service supply chain and smart contract information. Participants are required to transmit data to update the content and state of the contract and synchronize with the actual business. In addition, the smart contract of the logistics supply chain has built-in state attributes to match each link of the logistics service. After the logistics service status is updated, the contract status information will also be updated synchronously.

After the medical device smart contract change mechanism is added, the contract status will be synchronized with the logistics service status. The business processes of logistics companies will be recorded on smart contracts and blockchains in the form of state changes to achieve the effective integration of “logistics” and “information flow.” The construction of the smart contract model of the medical device service supply chain in the context of the blockchain is actually aiming at the shortest total order scheduling completion time, assigning the service operation to the logistics company and recording the start and end time of the operation in the blockchain. The proposed smart contract model is recorded on the blockchain in the form of code. When the conditions of the logistics service agreement become effective, the code will be automatically executed to complete the selection and scheduling of medical device logistics service providers.

The classic heuristic algorithm ant colony algorithm is used to solve the smart contract model, and the algorithm steps are shown in Figure 8. The ant colony algorithm uses the walking path of the ants to represent the feasible solution to the problem to be optimized. All paths of the entire ant colony constitute the solution space of the problem to be optimized. Ants with a shorter path release more pheromone. As time progresses, the accumulated pheromone concentration on the shorter path gradually increases, and the number of ants that choose this path increases. In the end, the entire ant will concentrate on the best path under the effect of positive feedback. At this time, it corresponds to the optimal solution of the problem to be optimized. The algorithm has good robustness.

The ant colony algorithm is used to select companies in the medical device scheduling service supply chain and coordinate the operations of each order to allocate the operations of scheduling each order to the companies that can provide services so that the order completion time is shortest. The basic idea is to let the ants schedule according to the corresponding service level information provided by the logistics enterprise and use the positive feedback characteristics of the ant colony algorithm to select the best feasible path for each order.

The effectiveness of the ant colony algorithm in the medical equipment logistics scheduling model is verified through experiments. The compilation environment uses PyCharm, the computer is configured as Inter (R) Core (TM) i5-7200, the main frequency is 2.50 GHz, and the installed and running memory is 8 GB.

## 3. Results

### 3.1. Performance Analysis of Medical Supplies Management Using Hyperledger Fabric Consensus Mechanism

When *n*=10, *λ*=0.4, the rate of change of hacker attacking nodes is shown in Figure 9:

In Figure 9, the probability of the attacker's success in control increases with the number of control nodes, but the trend is very flat. Only when the number of rules exceeds eight will the attack success rate be higher.

The security of the improved Hyperledger Fabric consensus mechanism is guaranteed and can be used.

The system security test result is shown in Figure 10:

In Figure 10, when more than half of the endorsing nodes are attacked for the original scheme, the attacker successfully manipulated all transactions. Under the condition of 10,000 transactions, the probability of an attacker with the optimized consensus mechanism successfully controlling the trade is only 7.2%.

Even if more than half of the endorsing nodes are attacked in the transaction after the optimized scheme is adopted, the optimized method can still run safely. The original consensus mechanism has completely fallen of fabric.

The results of the time spent on processing each transaction are shown in Figure 11:

In Figure 11, as the number of transactions increases, the transaction time gradually gets longer. The optimized solution is about 50% faster than the original solution in transaction processing speed.

In terms of transaction processing speed, the proposed optimization scheme has advantages.

The comparison result of transaction delay is shown in Figure 12:

In Figure 12, as the number of transactions increases for the two schemes, transaction delays increase accordingly. However, the more the number of transactions increases, the more pronounced the optimized solution optimization of the transaction delay. The optimization rate reaches 128% at the time of 1000 transactions. This is more than twice as high as before being optimized.

The proposed optimization scheme has advantages in the optimization of transaction delay. As the difficulty of the task increases, its benefits become more pronounced.

### 3.2. Performance Analysis of Smart Contract Model of Medical Equipment Dispatching Supply Chain

The impact of the smart contract model on the order completion time is compared with the performance of similar medical device scheduling algorithms in literature [24] and literature [25], as shown in Figure 13:

As Figure 13 suggests, the total time to complete the order of the medical device scheduling model with a smart contract is saved by 5 days compared with the historical service time of 19 days, and the efficiency is improved by 26.3%, which is better than the performance of similar medical device scheduling algorithms.

The use of intelligent contracts saves a great deal of time and cost for the medical device logistics scheduling supply chain and can form economic benefits with obvious advantages.

## 4. Conclusions

With the popularization of the innovation, experimentation of new technologies such as blockchain, and the popularization of applications in multiple fields, including supply chain management, blockchain technology still has advantages for the dispatch of medical supplies for emergency emergencies in the medical industry. The use of blockchain technology in the medical material platform can better realize the real-time sharing of information. The upstream and downstream of the supply chain can achieve effective and trustworthy mutual cooperation and establish a low-cost and high-efficiency medical material supply system. Through the research of blockchain technology, using the drawbacks of Fabric's original consensus mechanism, a medical material management network security scheduling scheme using the Hyperledger Fabric consensus mechanism has been established. Aiming at the particularity of medical devices in medical supplies, a medical device scheduling supply chain model using smart contracts has been established and its performance has been verified. The proposed scheduling scheme that incorporates supply chain technology has been verified in terms of security, transaction time, and the probability of being successfully attacked. The proposed schemes all show superior performance. Some shortcomings still exist: in the medical device scheduling problem, the punishment mechanism for companies submitting information that does not meet actual requirements is not considered. A penalty function can be added in future research to make the proposed scheme more in line with actual requirements.

## Figures and Tables

**Figure 1:** Block structure composition of Bitcoin.

**Figure 2:** Schematic diagram of Hyperledger Fabric consensus mechanism.

**Figure 3:** Schematic diagram of Hyperledger Fabric consensus mechanism.

**Figure 4:** Network topology diagram of the current medical material platform.

**Figure 5:** Network topology diagram of the expanded medical material platform.

**Figure 6:** The final network topology diagram of the medical supplies platform.

**Figure 7:** Smart contract model design in the context of blockchain.

**Figure 8:** Flow chart of ant colony algorithm.

**Figure 9:** Probability of successful attack.

**Figure 10:** Number of occurrences of a node without endorsement.

**Figure 11:** Comparison of transaction time between the two schemes.

**Figure 12:** Comparison of transaction delay between the two schemes.

**Figure 13:** Influence of whether to adopt smart contract model on order completion time.

## Data Availability

The dataset used to support the findings of this study is available from the corresponding author upon request.

## References

[1] Slagman A., Behringer W., Greiner F., Klein M., Weismann D. (2020). Medical emergencies during the COVID-19 pandemic: an analysis of emergency department data in Germany. *Deutsches Ärzteblatt International*.

[2] Al-Hassan M., AlQahtani S. (2019). Preparedness of dental clinics for medical emergencies in Riyadh, Saudi Arabia. *The Saudi dental journal*.

[3] Andoni M., Robu V., Flynn D. (2019). Blockchain technology in the energy sector: a systematic review of challenges and opportunities. *Renewable and Sustainable Energy Reviews*.

[4] Saberi S., Kouhizadeh M., Sarkis J., Shen L. (2019). Blockchain technology and its relationships to sustainable supply chain management. *International Journal of Production Research*.

[5] Min H. (2019). Blockchain technology for enhancing supply chain resilience. *Business Horizons*.

[6] Pan X., Pan X., Song M. (2020). Blockchain technology and enterprise operational capabilities: an empirical test. *International Journal of Information Management*.

[7] Sammeta N., Parthiban L. (2021). Hyperledger blockchain enabled secure medical record management with deep learning-based diagnosis model. *Complex & Intelligent Systems*.

[8] Ogundokun O., Awotunde J. B., Adeniyi E. A., Ayo F. E. (2021). Crypto-Stegno Based Model for Securing Medical Information on IOMT platform. *Multimedia Tools and Applications*.

[9] Garett R., Young S. D. (2021). The Potential Application of Blockchain Technology in HIV Research Clinical Practice, and Community Settings. *Health and Technology*.

[10] Janssen M., Weerakkody V., Ismagilova E., Irani Z. (2020). A framework for analysing blockchain technology adoption: integrating institutional, market and technical factors. *International Journal of Information Management*.

[11] Ali O., Ally M., Dwivedi Y. (2020). The state of play of blockchain technology in the financial services sector: a systematic literature review. *International Journal of Information Management*.

[12] Mohanta B. K., Jena D., Panda S. S., Sobhanayak S. (2019). Blockchain technology: a survey on applications and security privacy challenges. *Internet of Things*.

[13] Kouhizadeh M., Saberi S., Sarkis J. (2021). Blockchain technology and the sustainable supply chain: theoretically exploring adoption barriers. *International Journal of Production Economics*.

[14] Dutta P., Choi T. M., Somani S., Butala R. (2020). Blockchain technology in supply chain operations: applications, challenges and research opportunities. *Transportation Research Part E: Logistics and Transportation Review*.

[15] Wang Q., Su M. (2020). Integrating blockchain technology into the energy sector—from theory of blockchain to research and application of energy blockchain. *Computer Science Review*.

[16] Abu-Elezz I., Hassan A., Nazeemudeen A. (2020). The benefits and threats of blockchain technology in healthcare: a scoping review. *International Journal of Medical Informatics*.

[17] Zhou Q., Huang H., Zheng Z., Bian J. (2020). Solutions to scalability of blockchain: a survey. *IEEE Access*.

[18] Bodkhe U., Tanwar S., Parekh K. (2020). Blockchain for industry 4.0: a comprehensive review. *IEEE Access*.

[19] Nanayakkara S., Rodrigo M. N. N., Perera S., Weerasuriya G. T., Hijazi A. A. (2021). A methodology for selection of a Blockchain platform to develop an enterprise system. *Journal of Industrial Information Integration*.

[20] Xu X., Sun G., Luo L., Cao H. (2021). Latency performance modeling and analysis for hyperledger fabric blockchain network. *Information Processing & Management*.

[21] Gorenflo C., Lee S., Golab L., Keshav S. (2020). FastFabric: scaling hyperledger fabric to 20 000 transactions per second. *International Journal of Network Management*.

[22] Jiang L., Chang X., Liu Y., Misc V. B. (2020). Performance analysis of Hyperledger Fabric platform: a hierarchical model approach. *Peer-to-Peer Networking and Applications*.

[23] Mandl K. D., Gottlieb D., Mandel J. C., Jones J., Ellis A. (2020). Push button population health: the SMART/HL7 FHIR bulk data access application programming interface. *NPJ digital medicine*.

[24] Liu Q. (2020). Integrated deteriorating maintenance and patient scheduling for single medical device with heuristic algorithm. *international journal of bio-inspired computation*.

[25] Ozturk O. (2020). A bi-criteria optimization model for medical device sterilization. *Annals of Operations Research*.

